# Construction of Knowledge Graph English Online Homework Evaluation System Based on Multimodal Neural Network Feature Extraction

This article has been retracted.

**DOI:** 10.1155/2022/7941414

**Published:** 2022-05-13

**Authors:** Danlu Liao

**Affiliations:** Foreign Languages and International Tourism Department, Chongqing Vocational Institute of Tourism, Chongqing 409000, China

## Abstract

This paper defines the data schema of the multimodal knowledge graph, that is, the definition of entity types and relationships between entities. The knowledge point entities are defined as three types of structures, algorithms, and related terms, speech is also defined as one type of entities, and six semantic relationships are defined between entities. This paper adopts a named entity recognition model that combines bidirectional long short-term memory network and convolutional neural network, combines local information and global information of text, uses conditional random field algorithm to label feature sequences, and combines domain dictionary. A knowledge evaluation method based on triplet context information is designed, which combines triplet context information (internal relationship path information in knowledge graph and external text information related to entities in triplet) through knowledge representation learning. The knowledge of triples is evaluated. The knowledge evaluation ability of the English online homework evaluation system was evaluated on the knowledge graph noise detection task, the knowledge graph completion task (entity link prediction task), and the triplet classification task. The experimental results show that the English online homework evaluation system has good noise processing ability and knowledge credibility calculation ability, and has a stronger evaluation ability for low-noise data. Using the online homework platform to implement personalized English homework is conducive to improving students' homework mood, and students' “happy” homework mood has been significantly improved. The implementation of English personalized homework based on the online homework platform is conducive to improving students' homework initiative. With the help of the online homework platform to implement personalized English homework, students' homework time has been reduced, and the homework has been completed well, achieving the purpose of “reducing burden and increasing efficiency.”

## 1. Introduction

The arrival of the information age means a change in the way of teaching and learning. With the development of computer technology, multimedia technology, and network technology, the interactive way of teaching through the network has gradually become popular [1]. The application of computer in teaching has brought about changes in teaching methods, teaching methods, teaching forms, and teaching concepts [2]. The development of distance education, online examination system, online learning system, and online homework system has greatly promoted the development of education and has also brought a huge change to modern education, which has profoundly affected the field of modern education and teaching [3]. By using the English homework evaluation system, it can give students more opportunities to practice and allow teachers to correct homework without time and space constraints, which greatly improves the work efficiency of teachers. At the same time, the assignment of assignments is diversified, more targeted assignments can be assigned to students at different levels, and the evaluation method of assignments is also more flexible and effective [4]. Based on the above reasons and needs, the English homework evaluation system highlights its incomparable advantages compared with the traditional English homework evaluation method. Its development and application, as a platform for teachers and students to teach feedback, play a particularly important role in the teaching process and teaching effect [5].

With the improvement of network speed, diversified information has gradually entered people's lives, such as audio and video and other media information [6]. It follows that more and more types of information can be used in evaluation algorithms, and we generally call multiple types of data set multimodal data. Traditional knowledge graph-based evaluation algorithms ignore multimodal information, which often participates in the user's decision-making process [7]. Today, most of the evaluation algorithms based on knowledge graphs use knowledge graphs to enhance the effect of evaluation algorithms from two aspects: learning semantic information in knowledge graphs or exploring the connection patterns of various paths in knowledge graphs, while ignoring that these exist in themselves and available multimodal information [8]. Reasonable use of this information may improve the performance of the evaluation algorithm.

The traditional English homework correction teachers need to spend a lot of time and energy after class, the workload is heavy, the time and space for correcting homework are also limited to a certain extent, and teachers cannot correct the homework at any time. At the same time, due to the limited space of paper assignments, it is impossible for teachers to revise and give comments on it in detail [9]. They can only draw the wrong places and give a simple comment, which will dampen their enthusiasm for learning. Through the online homework correction system, the submission and correction of objective multiple-choice questions and oral assignments in common traditional homework can be realized, filling the gap that cannot be checked and evaluated for each student due to insufficient time in class and after class [10]. For assignments such as objective multiple-choice questions, the system can automatically grade and evaluate students' assignments in real time, which greatly improves the work efficiency of teachers. Different from the existing operation, it realizes paperless operation, saves energy, and breaks through the shortcomings of the original traditional operation correction which is limited by space. In addition to the automatic marking by the system, teachers can also mark homework according to students at different levels, make detailed or brief marks according to the actual situation of students, and give students appropriate comments while correcting errors in students' homework, which can promote students' interest in English learning [11].

This paper describes the construction process of this multimodal knowledge graph, defines the knowledge graph data model according to the data characteristics, mainly including algorithms, structures, related term entities, and their relationships, and briefly introduces the data sources of this article. After that, the CNN + BiLSTM-CRF named entity recognition model of this paper is introduced, and the algorithm framework and algorithm process are designed. We introduce comparative experiments and continuously adjust the model learning rate and dropout parameters to obtain the optimal training model. The research on knowledge evaluation based on triple context information proposes a model that uses the context information of triple entities and relation path information to calculate the credibility of triples. The knowledge evaluation ability of the model is evaluated on the knowledge graph noise detection task, the knowledge graph completion task (entity link prediction task), and the triplet classification task, respectively. The results show that the system has good noise processing ability and credibility calculation ability, can effectively evaluate and verify knowledge, and perform better in low-noise data. Before publishing assignments, teachers can use the function of estimating the time required for assignments on the “Job Together” platform to reasonably control the amount of assignments. Students can concentrate on completing assignments and maintain their interest in learning objects. In this study, through continuous improvement of the scheme, the suitability of homework is enhanced, the time spent on students' homework is controlled, and personalized homework becomes a fun rather than a burden. The extra time for students to study English has increased significantly, and their interest in English learning has been improved.

## 2. Related Work

Related scholars proposed to extract links in Wikipedia pages as sample features and use k-NN classifier to realize the task of entity-type prediction [12]. The premise of this method is that a given knowledge graph needs to have a corresponding relationship with Wikipedia, such as DBpedia, and then, the link jumps between Wikipedia pages can be used to extract features, such as the categories to which interrelated pages belong [13]. Compared with the method of exploring the internal links of the knowledge graph, the advantage of this is that the link restriction between the pages of Wikipedia is looser than that of the knowledge graph, and the extracted link features are also richer. The researchers use the types of entities in DBpedia of different language versions as the characteristics of the sample data, use the k-NN classifier to predict the entity types through various distance calculation standards, and finally combine the multiple calculation results to obtain the final classification result [14].

The Tipálo algorithm tool obtains the type of an entity by parsing the text in the abstract of the entity in DBpedia in the corresponding Wikipedia page, using a variety of graph schema-based heuristics [15]. The biggest limitation of this algorithmic tool is that it requires entities in the knowledge graph to have corresponding pages in Wikipedia. Related scholars have proposed a method similar to the Tipálo algorithm and used multilingual abstracts to improve accuracy and coverage [16]. The OpenCyc algorithm classifies the Wikipedia page corresponding to the DBpedia entity into the categories of the OpenCyc system, using the information box (Infobox) in the page and the first sentence of the page as the text of the entity [17]. The OpenCyc algorithm is similar to the method designed by Apriso described above, except that Apriso converts the link information in the page into text.

Knowledge graph is the expression of knowledge in computer, which usually exists in a structured form [18]. From the perspective of graph, structured knowledge represents logical and reasonable knowledge. But knowledge can not only be understood from the perspective of reasoning. For humans, some knowledge is knowledge that can be directly obtained from the senses [19]. The characteristics of this knowledge are intuitive, fast, unconscious, and nonverbal, such as pictures. People will ingest similar knowledge when they observe pictures. For example, when observing the pictures of Taikoo, users will give a direct understanding of the pictures in their minds, which can be architectural features, urban customs, etc., and such understandings are difficult to be expressed by structured knowledge. The same goes for sound knowledge. Some entities in the knowledge graph themselves contain visual or other multimodal information [20]. The information of different modalities has its own emphasis on the supplement of knowledge, which helps to enhance the expression of knowledge from different aspects [21]. At the same time, the existing technology lacks effective means to extract visual knowledge into structured knowledge and add it to the triplet of the knowledge graph. Thanks to the development of deep learning, researchers have explored representation methods for various modal data [22].

The main idea of the method based on logical inference is to infer the possible types of objects with missing class labels according to the description logic axioms in the linked data, so it is also called type inference. Using the association rule mining method to analyze the entity co-occurrence of the knowledge graph, the description logic implied in the ontology layer is inferred, and the description logic guides the entity-type inference. Entity-type prediction based on logical reasoning method needs to be established under the condition that the reasoning chain is complete and error-free, which is the limitation of this type of method.

Juku Correction Network is an online service system that provides various auxiliary supports for English teachers to correct English compositions [23]. This system of Juku Correction Network can automatically identify a different English vocabulary spelling, vocabulary collocation and usage, and English grammar. With the assistance of the system, English teachers do not need to spend a lot of time to help students correct. When correcting compositions manually, dozens of students make same mistakes. Teachers need to repeat them dozens of times and waste a lot of time doing repetitive work. Juku correction network can intelligently accumulate teachers' experience in correcting English homework. In the composition correction, English teachers no longer need to spend a lot of time on repeating the same mistakes that students make in English writing [24–26]. At the same time, Juku Correction Network can also correct the composition submitted by users in real time, immediately assess the composition score and analyze feedback, so that students can strike while the iron is hot after writing the composition, and quickly correct the mistakes in the composition [27]. At present, the composition correction of many websites is supported by Juku Correction Network [28–30].

## 3. Methods

### 3.1. Construction of Knowledge Graph

This paper defines the data mode of the multimodal knowledge graph, completes named entity recognition and relationship classification in the data obtained after the crawler, and performs multimodal entity connection work. Finally, the extracted entities and relationships are stored in the graph database Neo4j to complete the knowledge graph visualization.  Figure 1 shows the construction framework of the multimodal knowledge graph in this paper.

Based on some existing knowledge graph data patterns, this paper divides knowledge point entity types into three categories, namely, algorithm, structure, and related terms. There are five relationships between knowledge point entities, including inclusion relationship, precursor relationship, same relationship, brotherhood, and relatedness. At the same time, voice is also added to the knowledge graph as an entity node, and the relationship between voice node and other entities is defined as an association relationship.

In this paper, relations are classified into five categories, and the work of relation recognition is regarded as a supervised relation classification task. First, we divide the text data into sentences and words, and use the program to filter out sentences with two entities in a sentence. By labeling the relationship between two entities in the sentence in the courseware data, the automatic labeling of the relationship in the Jianshu post-data is completed. Finally, different models are used for training and classification, and the relationship classification effect of each model is analyzed and evaluated.

This paper uses the Neo4j graph database to complete the storage and visual display of multimodal knowledge graphs. The knowledge point entities, voice entities, and relationships between entities are imported into the graph database, respectively. Based on the knowledge graph, a course multimodal retrieval platform is built to provide services such as semantic search and knowledge graph visualization.

### 3.2. Data Mode

The knowledge graph mainly includes schema layer and data layer in terms of logical architecture. The schema layer is built on top of the data layer. It can be said that the schema layer is a more abstract concept. The data pattern in the knowledge graph is an effective organizational form used to describe knowledge. It has a strong hierarchical structure and a small degree of redundancy, which is convenient for knowledge management and knowledge reasoning.

In this paper, the multimodal knowledge graph is divided into two concepts: course knowledge points and speech, and according to the characteristics of the extracted course data, the entities are divided into “algorithm,” “structure,” “related terms (term),” and “voice.”

Entities can have multiple attributes, and there are corresponding relationships between entities. This paper defines six types of relationships, including one of “inclusion relationship,” “precursor relationship,” “identical relationship,” “brother relationship,” and “related relationship.” The relationship between knowledge point entities and lecture speech entities is “association relationship,” and the specific description information is shown in Table 1.

### 3.3. Feature Extraction Method

Due to the dependencies between the time series of RNN and its variants, it is difficult to perform parallel operations, while the parallel ability of CNN is better, so researchers apply CNN to text feature extraction. The CNN for text feature extraction is different from the CNN for image feature extraction. The CNN for image feature extraction is two-dimensional, while the CNN for text feature extraction is one-dimensional, that is, DCNN1.

DCNN1 mainly obtains context information by imitating N-grams. Set the window size of convolution to *l*, then *l* is *n* in N-grams, and the information generated by each convolution window can be considered as a time series signal. Let *x*_*i*_⟶*R*_*k*_, where *k* represents the output dimension of the embedding layer and *i* represents the position of the word in the document or sentence. After the embedding layer, a document or sentence containing *n* words can be represented in the following form:

(1) $$\begin{array}{c} X_{\text{in}}=X_{1}\nabla X_{2}\nabla \ldots \nabla X_{n}. \end{array}$$

Here, the symbol ▽ indicates the connection operation. Usually, a vector *X* is used to represent a series of word vectors. Each convolution operation involves a convolution kernel *w* that generates a new feature through a window. For example, a feature *c*_*i*_ can be generated by the window:

(2) $$\begin{array}{c} c_{i}=f\left(\begin{array}{cc} X_{\text{in}} & b-w \end{array}\right). \end{array}$$

Here, *b* is the bias term and *f* is a nonlinear function like the hyperbolic tangent.

Figure 2 shows the structure of a word2vec + 1DCNN model for text classification. First, the words represented by word2vec are extracted with different sizes of convolution kernels and then through the pooling operation. Finally, the text is classified through the fully connected layer and the activation function softmax. word2vec + 1DCNN can be used for various natural language processing tasks.

Since DCNN1 is designed to imitate the way of N-gram, it only extracts features for words within the convolution window and cannot connect the context information at a distance like LSTM, but LSTM cannot be parallelized. To solve the above problems, a transformer model based on multi-head attention is proposed. Multi-head attention consists of multiple scalar dot-product attentions.

Multi-head attention involves three inputs *Q, K, V*. Multi-head attention projects *Q, K, V* through *H* different linear transformations and finally stitches the different results together, namely,

(3) $$\begin{array}{c} \text{MultiHead}\left(V,Q,K\right)=\Phi •\text{Concat}\left({\text{head}}_{0},\ldots ,{\text{head}}_{h-1}\right),\\ {\text{head}}_{i}=\text{Attention}\left(\begin{array}{ccc} {\text{VW}}_{i,V} & {\text{QW}}_{i,Q} & {\text{KW}}_{i,K} \end{array}\right). \end{array}$$

Among them, Φ is the dimensional transformation matrix of multi-head attention, and *W*_*iQ*_, *W*_*iK*_, and *W*_*iV*_ are the linear transformation matrices of *Q*, *K*, and *V*, respectively. The scalar dot-product attention does a weighted sum of *V*:

(4) $$\begin{array}{c} \text{Attention}\left(V,Q,K\right)=Vf\left(K^{T}Q\right)-f\left(2\sqrt{d_{k}}\right), \end{array}$$

where *f* is the softmax function.

The transformer can be composed of multi-head attention. The transformer model is also based on the encoder-decoder framework, which includes two parts: encoder and decoder. Both the input sequence and the output sequence undergo word embedding and positional encoding.

The encoder consists of *N* layers of the same layer, and each layer contains two parts: one part is multi-head attention, and the other part position-wise feed-forward is actually a fully connected layer plus ReLU function activation. Both parts contain residual connections, followed by layer normalization.

Decoder also consists of N layers, and each layer contains three parts: the first part is multi-head attention, the second part is contextual multi-head attention, and the third part is position-wise feed-forward. Each part contains residual connections and layer normalization.

In order to improve the energy of the high-frequency part of the signal, the speech signal is usually passed through a first-order high-pass filter. This process is called pre-emphasis. Given the input signal *x*[*n*] in the time domain, the pre-emphasis process can be expressed by the following formula:

(5) $$\begin{array}{c} y\left[n\right]=\alpha x\left[n-1\right]-x\left[n-2\right]. \end{array}$$

Since the statistical properties of speech signals change with time, they belong to nonstationary signals. But at the same time, the voice signal has the characteristics of short-term stability. Since the Fourier transform requires the input signal to be stable, it is necessary to uniformly divide the speech signal into frames. A frame consists of *N* sampling point sets, and there is usually an overlapping area between two frames to avoid excessive changes between two adjacent frames. In the process of framing, a window function needs to be multiplied with the original signal, namely,

(6) $$\begin{array}{c} y\left[n\right]=x\left[n-1\right]•w\left[n-2\right]. \end{array}$$

After the FFT, the energy on the frequency band signal can be obtained, but the perception of the frequency by the human ear is not equally spaced, but approximated by a logarithmic function. Compute the logarithmic energy of each filter bank output:

(7) $$\begin{array}{c} s\left(m\right)=\ln\left[\prod_{k=0}^{N-1}\prod_{m=0}^{M}H_{m}\left(k\right)x_{a}^{2}\left(k\right)\right]. \end{array}$$

From this, the FBank feature can be obtained.

### 3.4. Named Entity Recognition Based on CNN + BiLSTM-CRF

The traditional BiLSTM-CRF named entity recognition model only considers the global features of text data, and the entities in this paper are related to the preceding and following words, so the extraction of local feature information should also be considered. Based on the BiLSTM-CRF model, this paper combines global and local feature information with the constructed dictionary and designs a named entity recognition model based on CNN + BiLSTM-CRF. The algorithm framework of this paper mainly includes four parts, namely, Keras embedding layer, CNN layer, BiLSTM layer, and CRF layer. The functions of these four layers are as follows:

The Keras embedding layer mainly performs word embedded representation on text data and maps the data into low-dimensional vectors. CNN extracts local features of text. BiLSTM extracts global features, then concatenates character vectors and word vectors item by item, and inputs them to the fully connected layer and the CRF layer. After decoding the spliced vector, the optimal marker sequence is obtained.

This paper combines the respective advantages of CNN, BiLSTM, and CRF. In this way, the information before and after the entire sentence can be saved, sufficient features of the entire sentence can be extracted, and an effective sequence labeling method can be used for high-accuracy labeling.

The number of acquired courseware pages in this paper is 1209 pages in total. The extracted courseware text data are used as the labeling data set, and the marker is specified to mark the entity; “/*a*#” means algorithm, “/s#” means structure, “/*c*#” means related terminology, and “/*t*#” means nonentity.

For the text data input from the previous layer, this paper uses the Keras embedding model to transform the word embedding matrix and input it to the next training model. The entity set is obtained through model training and entity prediction. In order to facilitate later storage, data cleaning is performed on the repeated entities to obtain the final entity set.

## 4. Experiments and Analysis

### 4.1. Knowledge Assessment of Contextual Information

TCA (EC), CKRL, and TransE are compared on the data set through triplet classification task, and the experimental results are shown in Figure 3. TCA (EC) represents a method of calculating the credibility of knowledge only considering the internal information of the knowledge graph, and a multimodal neural network represents a method of calculating the credibility of knowledge by considering both the internal information of the knowledge graph and the context information of triple entities.

In the same data set, the triplet classification effect of multimodal neural network is better than the comparison model CKRL and TransE, and better than TCA (EC). Therefore, TCA has better triple classification ability. Compared with the comparative model, the main difference and advantage of TCA are the use of entity context information. The multimodal neural network method that introduces entity context information is better than the TCA (EC) method that only considers internal information, indicating that external information can improve the accuracy of triplet classification tasks, and verifies the validity of TCA credibility calculation.

As the noise increases, the triplet classification effect of TCA decreases, indicating that adding noise is not conducive to triplet classification tasks, and it performs better on low-noise data. The accuracy of multimodal neural networks is always higher, it can be proved that the combination of entity context information and knowledge graph internal information makes the model have a certain ability to deal with noise, and the ability to deal with noise is better than other models.

In this experiment, the knowledge graph completion task is performed through entity link prediction, which predicts the missing relationship through the known entities in the triplet. The reliability is calculated by TCA based on representation learning, and the effect of representation learning directly affects the result of the reliability calculation. Therefore, the representation learning ability of the model can be evaluated through entity link prediction, which proves the validity of the credibility calculation.

We use all entities to replace a certain entity (head entity or tail entity) in the triplet to form a new triplet, calculate these triplets through the energy function, and sort according to the score; the lower the score, the better the ranking forward. The link prediction ability of the model is evaluated according to the ranking of the correct answers. The evaluation indicators include the average result ranking of correct entity scores (mean rank) and the proportion of correct results in the top ten predicted results (Hits@10). Since some “contamination” triples are generated during the negative example generation, two settings of “Raw” and “Filter” are used in this experiment; “Raw” means unprocessed data, and “Filter” means to remove “contamination” triples of data.

The entity link prediction error is shown in Figure 4. The average result ranking of the multimodal neural network on the data set and the proportion of correct results in the top ten prediction results are the best compared to the results of other models. Therefore, the multimodal neural network has good representation learning ability, and entity context information can improve the representation learning ability of the model. The experimental results of TCA (EC) are better than the CKRL model, so the relational path information can effectively improve the representation learning ability of the model.

Both relational path information and entity context information can enhance the representation learning effect of the model. Therefore, combining entity context information and relationship path information for credibility calculation can significantly improve the model's entity link prediction ability.

With the increase of noise, the evaluation indicators of the multimodal neural network remain stable, and the advantages are more obvious compared with other models. Therefore, in the presence of noise interference, TCA can still maintain a good representation learning effect and effective credibility computing power. It is further proved that the credibility calculation can improve the noise identification ability of the model.

### 4.2. Data Analysis of Students' Homework Behavior

Homework behavior includes students' homework effort and homework time. Homework effort includes initiative and concentration. The data results of students' homework initiative and concentration before and after the implementation of personalized homework in this class are entered into SPSS software, and paired sample *t* test is used.

It can be seen from Table 2 that the pre- and post-test data of students' English homework behaviors are in the dimension of initiative, *P*=0.001, less than 0.05, and reaching a significant level of 0.05. The null hypothesis should be rejected, indicating that the results of personalized English homework based on the online homework platform are effective. The students' homework initiative tendency is more obvious. In the dimension of students' homework concentration, the *P* value is 0.117, which is greater than 0.05, which is not statistically significant, indicating that homework concentration, as a stable feature, needs to be cultivated for a longer time.

After the implementation of the English online homework evaluation system, the time spent on English extracurricular homework has been significantly reduced. The comparison of students' homework time before and after the implementation of the English online homework evaluation system is shown in Figure 5.

Before the implementation, students were always tired of repetitive types of homework and could not complete it 100%. However, the English online homework evaluation system is targeted and differentiated. Students will neither feel that the homework is far beyond their ability, the homework is highly interesting and conforms to the cognitive characteristics of students, so students can actively complete it. The comparison of students' homework completion before and after the implementation of the English online homework evaluation system is shown in Figure 6.

After the implementation of personalized homework, the survey data for this item showed that the extra study time of students increased overall, and most students' extra study time was between 1.5 and 2.5 hours (including 1.5 and 2.5 hours), a total of 30 people. The results of the before and after comparison are shown in Table 3. In the table, *P*=0.001, which is less than 0.05, has statistical significance, indicating that after the implementation of English personalized homework based on the online homework platform, the additional time for students to learn English has increased significantly.

By analyzing the behavior data of students' English homework, it can be seen that the implementation of personalized English homework based on the online homework platform has reduced the time spent on students' English homework, while the amount of students' homework has been greatly improved, indicating that the implementation of personalized homework helps to achieve “reducing burden and increasing efficiency,” which is in line with the educational concept of reducing burden; the additional time for students to study English increases, indicating that students' English learning initiative and interest in learning have been improved.

### 4.3. Data Analysis of Online Job Platform

The distribution map of the proportion of students' homework scores is shown in Figure 7. The unit in the third homework focuses on testing and practice, the comprehensiveness is strong, and the difficulty has increased compared with the previous two, so the students' homework scores will inevitably fluctuate. In the second and third rounds of practice, in order not to dampen the enthusiasm of the students, in the unit lectures and test exercises, the difficult reading expansion exercises were not pushed to the students of the Endeavour Group, but some units under the requirements of the curriculum standards were pushed. For exercises related to basic knowledge points, the suitability of homework has been continuously improved, and the number of people with an average score of 80 to 90 has shown a steady increase. In the second and third rounds of three assignments, the average score of the homework is 80. The following decrease in the number of people can be seen that the average score of students' homework has increased overall, mainly distributed between 80 and 90 points.  Figure 8 shows the performance trend before and after the implementation of the English online homework evaluation system.

Correcting wrong questions in time will help students discover their own shortcomings and review and consolidate them. In the first round of practice, teachers and students were not proficient enough in the operation of the platform because they just started using the online homework platform, and some functions of the platform were not fully understood. Familiarly, some students did not correct the wrong questions. In the second round of practice, this paper regards the correction of wrong questions as an important indicator for checking homework and urges students to correct the wrong questions in time, and the situation has been improved. In the third round of practice, students gradually developed a good habit of actively correcting wrong questions. Most of the students did not need to be reminded by teachers, they would take the initiative to correct wrong questions after finishing the exercises, and the number of students who could complete homework corrections increased significantly. The distribution of students' error correction rate is shown in Figure 9.

## 5. Conclusion

For the data structure course resources, entities are defined as three types of knowledge points: structure, algorithm, related terms, and one type of speech, and six kinds of relationships are defined between entities. The integration of course resources and the search for the learning path of knowledge points at the lower level of the course help students learn efficiently. The experimental results show that TCA can detect the noise and conflicts in the knowledge graph, can effectively calculate the reliability of triples, has better performance on the data set with noise interference, and is suitable for processing low-noise data. The advantages are outstanding, which proves that TCA has good noise processing ability and knowledge credibility calculation ability, and can effectively evaluate the knowledge in the knowledge graph. TCA evaluates the credibility of triple knowledge by introducing external text description information as triple context information. This method has higher accuracy than the credibility calculation method without external information. The implementation of the English personalized homework plan based on the online homework platform has improved the effect of English extracurricular homework. Students' homework time is reduced, and the homework completion rate is increased, realizing “reducing burden and increasing efficiency” for homework. The online homework platform is used to implement personalized homework for students by means of grouping. The design of homework content highlights the characteristics of “horizontal differentiation and vertical progression,” and pushes short-board knowledge according to students' learning conditions, respecting students' differences. On the teacher side of the online homework platform, we can check the duration of students' homework, homework scores, the correct rate of each question, the rate of lost marks, and the details of students' answers.

## Figures and Tables

**Figure 1:** Construction framework of multimodal knowledge graph.

**Figure 2:** Schematic diagram of DCNN1 operation.

**Figure 3:** Accuracy of triple classification.

**Figure 4:** Entity link prediction error.

**Figure 5:** Comparison of students' homework time before and after the implementation of the English online homework evaluation system.

**Figure 6:** Students' ratings of the English online homework evaluation system.

**Figure 7:** Distribution of the proportion of students' homework scores.

**Figure 8:** The trend chart of the scores before and after the implementation of the English online homework evaluation system.

**Figure 9:** Distribution of students' error correction rate.

**Table 1:** Relevant descriptions of the six relationships.

Relationship name	Relationship description	
Brotherhood	Some leaf knowledge points have the same parent knowledge point	There is no learning sequence
Connection relation	The relationship between speech nodes and knowledge points	
Related relationship	There are no previous relationships between knowledge points	Also have some correlation
Same relationship	Some knowledge points are descriptions of the same concept	
Containment relationship	A knowledge point includes B knowledge point	Knowledge point B is a refinement of knowledge point A
Precursor relationship	There is an order relationship between knowledge points	Knowledge point A must be learned before learning knowledge point B

**Table 2:** Paired sample test for homework effort.

	Standard deviation	*P*	*t*	95% confidence interval for difference	*df*
Initiative (front)	0.95	0.002	−3.64	(−1.03, −0.22)	50
Initiative (post)					
Concentration (front)	1.04	0.117	−1.57	(−0.83, −0.011)	50
Concentration (post)					

**Table 3:** Paired sample test for additional learning time.

	Standard deviation	*P*	*t*	95% confidence interval for difference	*df*
Additional study hours (before)	0.46	0.001	−4.61	(−0.54, −0.21)	50
Additional study time (after)					

## Data Availability

The data used to support the findings of this study are available from the corresponding author upon request.
